# The High Expression of PTPRH Is Associated with Poor Prognosis of Human Lung Adenocarcinoma

**DOI:** 10.1155/2021/9932088

**Published:** 2021-07-29

**Authors:** Aifeng Chen, Shibiao Ding, Xiaoqiang Shen, Xuai Lin

**Affiliations:** ^1^Department of Respiratory Medicine, Affiliated Hangzhou Chest Hospital, Zhejiang University School of Medicine, Hangzhou 310058, China; ^2^Department of Clinical Laboratory, Affiliated Hangzhou Chest Hospital, Zhejiang University School of Medicine, Hangzhou 310058, China; ^3^Department of Medical Microbiology and Parasitology, and Department of Infectious Diseases, Affiliated Children's Hospital, Zhejiang University School of Medicine, 866 Yuhangtang Road, Hangzhou 310058, China

## Abstract

**Objective:**

The aim of the study is to explore the prognosis value of PTPRH in patients with lung adenocarcinoma (LUAD).

**Methods:**

Oncomine, UALCAN, and GEPIA databases were employed to examine the differential expression of PTPRH between LUAD and adjacent tissues. 100 pairs of LUAD and adjacent tissue samples were involved in this study. qRT-PCR and immunohistochemical staining were performed. Meanwhile, we analyzed The Cancer Genome Atlas (TCGA) data to investigate the correlation between PTPRH gene expression and clinicopathological characteristics. Kaplan-Meier analysis and univariate and multivariate Cox analyses were performed to estimate the relationship between PTPRH expression and LUAD prognosis. The evaluation performance was verified by drawing a ROC curve. In addition, through GSEA, the changes of PTPRH expression were analyzed by GSEA to screen out primarily affected signaling pathway.

**Results:**

Oncomine, UALCAN, and GEPIA databases showed that the mRNA expression of PTPRH in LUAD tissues was significantly higher than that in adjacent tissues. qRT-PCR and immunohistochemical staining indicated the mRNA and protein levels of PTPRH in LUAD tissues were markedly upregulated. TCGA data showed that the expression of PTPRH was significantly correlated with T stage and disease stage. Kaplan-Meier analysis showed that the patients with high PTPRH expression had a poor prognosis. Univariate and multivariate Cox analyses exhibited that PTPRH expression could act as an independent prognostic factor for LUAD. The ROC curve showed that PTPRH combined with various clinicopathological features could effectively predict the prognosis of LUAD. Finally, GSEA indicated that changes in PTPRH expression level may affect p53, VEGF, Notch, and mTOR cancer-related signaling pathways.

**Conclusion:**

Our results demonstrated that PTPRH was highly expressed in LUAD and may be closely correlated with the poor prognosis of LUAD patients.

## 1. Introduction

Lung cancer ranks first in both incidence and mortality and is the major health concern worldwide [1]. Lung adenocarcinoma (LUAD) is the most common type and is predicted to take 40% of all lung cancer cases [2, 3]. Patients diagnosed in the early stage of lung cancer can be treated with surgery and adjuvant therapy, yet the treatment often fails due to local or metastatic recurrence [4], leading to the 5-year survival rate of LUAD patients less than 15% [5]. Therefore, it is warranted to develop a novel therapeutic strategy for LUAD. The method based on molecular characterization has been reported to have a broad prospect in improving diagnostic accuracy and predicting therapeutic response [6], which makes the identification of effective biomarkers for cancer prognosis and diagnosis a hot topic for current studies.

PTPRH is known as stomach cancer-associated protein tyrosine phosphatase 1 (SAP-1), and it is also a receptor-type protein tyrosine phosphatase that locates specifically at microvilli of the brush border in gastrointestinal epithelial cells [7]. PTPRH is considered to be a negative regulator of integrin-mediated signaling which inhibits the integrin signaling by mediating the dephosphorylation of proteins associated with focal adhesion [8, 9]. PTPRH was differentially expressed in different cancers. Zhang et al. proved that PTPRH was highly expressed in epithelial ovarian cancer by using two independent gene expression datasets GSE44104 and GSE30274 [10]. Bujko et al. reported that PTPRH was downregulated in colorectal cancer, and its expression was epigenetically regulated by DNA methylation and chromatin modification [11]. Nagano et al. found that PTPRH was downregulated in the dedifferentiation process of human hepatocellular carcinoma, which may play a causal role in the progression of disease [8]. These findings reveal that PTPRH expression has tumor specificity. However, the expression and prognostic significance of PTPRH in LUAD remain largely unclear, which are worthy of further studying.

In this study, bioinformatics method was used to predict the expression of PTPRH in LUAD, while immunohistochemistry and qRT-PCR were performed to verify the expression of PTPRH in LUAD. Meanwhile, the correlation between PTPRH expression and clinicopathologic parameters was evaluated, and univariate and multivariate Cox analyses were employed to elucidate the potential effect of PTPRH on the prognosis of LUAD. Our study may provide a novel biomarker for the effective prognosis of LUAD.

## 2. Materials and Methods

### 2.1. TCGA Data Acquisition

The complete clinical information of 477 patients with LUAD was obtained from TCGA-LUAD dataset (https://portal.gdc.cancer.gov/). Patients were divided into the high-expression and low-expression groups according to the median of PTPRH expression.

### 2.2. Oncomine Analysis

The datasets of PTPRH mRNA expression level and DNA copy number in LUAD from multiple studies (Bhattacharjee Lung, Hou Lung, Landi Lung, Selamat Lung, Okayama Lung, TCGA Lung 2, and Weiss Lung) were analyzed using Oncomine database (https://www.oncomine.org/resource/login.html).

### 2.3. GEPIA

GEPIA (Gene Expression Profiling Interactive Analysis) database (http://gepia.cancer-pku.cn/) was employed to analyze the expression of PTPRH in normal lung and LUAD tissues. Based on TCGA and GTEx data, GEPIA can provide fast and customizable functionalities including differential expression analysis, profiling plotting, correlation analysis, patient survival analysis, similar gene detection, and dimensionality reduction analysis [12]. Thus, GEPIA was utilized to carry out survival analysis of patients with LUAD based on the expression of PTPRH.

### 2.4. UALCAN Analysis

According to clinical features like age, gender, cancer stage, and N stage, UALCAN (http://ualcan.path.uab.edu/index.html) is used to analyze the relative gene expression in tumor and normal tissue samples as well as in different tumor subgroups [13]. Here, we introduced *t*-test on the PTPRH transcripts in the subgroups (gender, age, and other parameters) of LUAD patients using UALCAN website.

### 2.5. Construction of Prediction Model and GSEA

Cox proportional risk regression model was used for univariate and multivariate analyses of prognostic factors. ROC curve was plotted to determine the specificity and sensitivity of the prognostic scoring based on PTPRH expression and clinicopathological features. GSEA software (http://www.gsea-msigdb.org/gsea/index.jsp) was utilized to perform GSEA of differential genes in the high- and low-expression groups of PTPRH, and FDR < 0.25 was used as the criterion for evident enrichment of the pathway.

### 2.6. Patients and Tissue Samples

A total of 100 pairs of LUAD and adjacent tissue samples were collected from patients who underwent surgical resection in Hangzhou Red Cross Hospital from June 2018 to October 2019. All samples were immediately frozen in liquid nitrogen. According to histopathological evaluation, the excised samples were identified as LUAD samples, and the adjacent nontumor tissues were 5 cm away from LUAD tissue margin. All patients never received preoperative chemotherapy or radiotherapy. Tumor staging was performed according to the TNM classification of malignant tumors provided by the Union for International Cancer Control. Our study was approved by the Ethics Committee of Hangzhou Red Cross Hospital and agreed by all the patients.

### 2.7. qRT-PCR

According to the manufacturer's protocol, total RNA was extracted from tissue samples by using Trizol (Invitrogen, Carlsbad, CA) and then converted to cDNA by PrimeScript RT-PCR reagent kit (Takara, Japan). Quantitative analysis was performed on ABI 7500 Real-Time PCR system (Applied Biosystems, USA) using SYBR Green Master Mix (Takara, Japan). Primer sequences are shown below: PTPRH: forward primer: GGCGGCACAACAGAGACTC, reverse primer: CTGTGGCAGTAGTGACAGTCC; GAPDH: forward primer: GGAGCGAGATCCCTCCAAAAT, reverse primer: GGCTGTTGTCATACTTCTCATGG. The relative expression of PTPRH was quantified by using the 2^-*Δ∆*Ct^ method. The experiment was conducted in triplicate.

### 2.8. Immunohistochemistry (IHC)

Tissue samples were fixed with formalin and embedded in paraffin and then cut into 5 *μ*m sections. Sections were subjected to antigen recovery with 10 mmol/L of citrate loading buffer (pH 6.0) in a microwave oven. After being washed three times with phosphate-buffered saline (PBS), the sections were incubated in 3% H_2_O_2_ for 20 min. After treatment with 10% goat serum albumin for 30 min, the sections were incubated overnight with rabbit polyclonal antibody PTPRH (5-20 *μ*g/ml, ab231727, Abcam, Cambridge, UK) at 4°C, followed by secondary antibody goat anti-rabbit IgG (1 : 2000, ab205718, Abcam, Cambridge, UK) at room temperature for 1 h. After being rinsed with PBS, the sections were then exposed to 3, 3′-diaminobenzidine (DAB) for color development and hematoxylin was used for counterstaining. Negative control sections were similarly processed, except that the primary antibody was replaced by normal rabbit serum. The experiment was conducted in triplicate.

### 2.9. Statistical Analysis

SPSS 22.0 (IBM Corp. Armonk, NY, USA) and GraphPad Prism 6.0 (GraphPad Inc., San Diego, CA, USA) were employed for statistical analysis. The chi-square test was used to evaluate the association between PTPRH expression and clinicopathologic parameters. *P* < 0.05 was considered statistically significant, and *P* < 0.01 was considered extremely significant.

## 3. Results

### 3.1. PTPRH Is Highly Expressed in LUAD

The PTPRH mRNA expression levels and DNA copy numbers in LUAD from multiple studies were analyzed based on Oncomine database, and the results indicated that the mRNA expression of PTPRH in LUAD tissues was notably higher than that in normal tissues (Figures 1(a)–1(f)), while there was no significant difference in PTPRH copy numbers between LUAD and normal tissues. GEPIA database was utilized to analyze the expression of PTPRH in LUAD and normal samples, in which the results were consistent with the analysis in Oncomine database (Figure 1(g)). Moreover, qRT-PCR was performed, finding that the expression of PTPRH in 100 LUAD tissue samples was significantly higher than that in paired adjacent tissues (Figure 1(h)). Similarly, the protein expression of PTPRH was found to be markedly upregulated in LUAD tissues by immunohistochemical staining (Figure 1(i)). Using UALCAN database, we analyzed the PTPRH transcripts in the normal group and LUAD subgroups classified by age, gender, disease stage, and N stage. The results indicated that the PTPRH expression levels of LUAD groups (except for group N3) were significantly higher than those of the normal group, and there was no significant difference between LUAD groups (Figures 2(a)–2(d)). Taken together, PTPRH was highly expressed in LUAD.

### 3.2. Association between PTPRH Expression and Clinicopathologic Features of LUAD

To determine the correlation between PTPRH expression and clinical factors in LUAD, clinical data of 477 LUAD cases were obtained from TCGA database, and two cases with incomplete clinical information were excluded. The association between PTPRH gene expression and clinicopathological features such as age, gender, T stage, and N stage of the rest 475 cases was analyzed. We found that there were significant differences in the distributions of T stage and pathological stage between the high-PTPRH group and low-PTPRH group (Table 1).

### 3.3. PTPRH Can Be Used as an Independent Prognostic Factor for LUAD

To investigate whether PTPRH expression could predict the survival status of LUAD, 477 cases obtained from TCGA database were divided into high- and low-expression groups based on PTPRH expression analyzed in GEPIA, and the association between PTPRH expression and overall survival (OS) was evaluated by the Kaplan-Meier survival curve. These findings suggested that the survival rate of patients with high PTPRH expression was remarkably lower than that of patients with low PTPRH expression (Figure 3(a)). To further determine the potential prognostic significance of PTPRH in LUAD patients, univariate Cox analysis was performed for PTPRH combining traditional clinicopathologic factors. As Table 2 illustrated, T stage, degree of lymph node metastasis, disease stage, and PTPRH expression were considered as high-risk factors, and they were significantly correlated with poor OS of patients with LUAD (*P* < 0.05). These high-risk factors were then subjected to multivariate Cox analysis, and it was found that disease stage and PTPRH expression were significantly related to prognosis of patients (*P* < 0.05), suggesting that they could be the independent prognostic factors for LUAD (Table 3). ROC curve was implemented to further verify the effect of PTPRH expression and clinicopathological features in predicting 3-year survival, and the AUC values of PTPRH, tumor stage, T, N, and combination of PTPRH and clinicopathological features were 0.616, 0.676, 0.605, 0.645, and 0.707, respectively (Figure 3(b)). To sum up, we believed that PTPRH combined with clinicopathological features could be used for the accurate prediction of LUAD prognosis.

### 3.4. GSEA

In order to further explore the signaling pathways involved in PTPRH in LUAD, we performed GSEA on PTPRH. As revealed by the results, changes in the expression of PTPRH in LUAD may affect VEGF (Figure 4(a)), Notch (Figure 4(b)), P53 (Figure 4(c)), and MTOR signaling pathways (Figure 4(d)).

## 4. Discussion

The occurrence of LUAD is associated with genetic factors, environmental factors, and other external factors (including smoking), among which genetic factors can be used as more objective biomarkers or indicators for diagnosis, treatment, and prognosis of LUAD [14]. The continuous development of high-throughput sequencing technology and database provides great convenience for verification of these biomarkers. Up to now, by analyzing different databases, several potential independent prognostic factors of LUAD have been screened, including BRMS1 [15], KIF18A [16], ERR*α* [17], and BSG [18]. However, there is still a lack of uniform standard for prognosis, and it is of urgent need to identify the biomarkers with better diagnostic and prognostic potential [17].

In this study, we first detected the mRNA expression level of PTPRH in various subtype datasets of LUAD by using Oncomine database, from which we found that the mRNA expression of PTPRH in LUAD tissues was significantly higher than that in normal tissues. The mRNA expression level of PTPRH in LUAD was further evaluated by GEPIA database, finding that PTPRH was upregulated in LUAD. Based on subgroup analysis across age, gender, disease stage, and N stage, the transcription level of PTPRH in LUAD patients was markedly higher than that in healthy persons. In addition, the protein and mRNA expression of PTPRH in clinical tissues was detected by using immunohistochemistry and qRT-PCR, respectively, and PTPRH was found to be highly expressed in LUAD, which was consistent with the results in epithelial ovarian cancer [10] and pancreatic cancer cell [19]. Moreover, PTPRH has been reported to regulate the intestinal tumorigenesis in mice [20]. In addition, another report showed that PTPRH is regulated by epigenetic DNA hypomethylation and is associated with prognosis in patients with non-small-cell lung cancer [21]. Therefore, we speculated that PTPRH may play an essential role in the development of LUAD.

To evaluate the effect of PTPRH on LUAD, we analyzed the association between PTPRH expression and clinicopathologic features such as age, gender, and TNM stage. PTPRH expression was found to be considerably related to T stage and disease stage. Previous studies have identified a 10-gene risk model composed of PTPRH and other nine genes, which performs well in predicting prognosis of LUAD patients [22]. In this study, the results of survival analysis revealed that patients with high PTPRH expression exhibited a remarkable decrease in OS. Univariate and multivariate Cox analyses further confirmed that PTPRH could be used as an independent indicator for LUAD prognosis.

In brief, our study validated that PTPRH was highly expressed in LUAD, and its expression was significantly correlated with T stage and disease stage. Patients with high PTPRH expression exhibited a remarkable decrease in OS, and PTPRH could be used as a biomarker for prognosis of LUAD. These findings not only provide useful clues for the determination of novel therapeutic targets in LUAD but also lay a foundation for the exploration of potential mechanisms of PTPRH in LUAD.

## Figures and Tables

**Figure 1:** The transcription and expression levels of PTPRH in LUAD. The mRNA expression level of Hou Lung (a), Landi Lung (b), Selamat Lung (c), and Okayama Lung (d) (1 for lung, 2 for lung adenocarcinoma); the copy number of PTPRH in TCGA Lung 2 (e) and Weiss Lung (f) (1 for blood, 2 for lung, and 3 for lung adenocarcinoma); (g) the mRNA expression of PTPRH in LUAD (red) and normal (black) tissues in GEPIA database; (h) the mRNA expression level of PTPRH in clinical LUAD tissues and paired adjacent tissues was detected by qRT-PCR; (i)the protein expression level of PTPRH in LUAD tissues and adjacent tissues was assessed by IHC (magnification 200x); ∗ means *P* < 0.05.

**Figure 2:** PTPRH transcription in normal lung tissues and LUAD tissues of different subgroups: (a) the relative expression of PTPRH in healthy individuals and in LUAD patients with different ages; (b) the relative expression of PTPRH in healthy individuals and male or female patients with LUAD; (c) the relative expression of PTPRH in healthy individuals and patients with different disease stages of LUAD; (d) the relative expression of PTPRH in healthy individuals and patients with different N stages of LUAD; ^∗^*P* < 0.05 and ^∗∗^*P* < 0.01.

**Figure 3:** PTPRH can act as an independent prognostic factor for LUAD. (a) Kaplan-Meier curve showed the OS in patients with high and low PTPRH expression. (b) The specificity and sensitivity of PTPRH expression and clinicopathological features in predicting 3-year survival were determined by plotting the ROC curve.

**Figure 4:** GSEA. GSEA shows that PTPRH expression mainly affects the (a) VEGF signaling pathway, (b) Notch signaling pathway, (c) P53 signaling pathway, and (d) mTOR signaling pathway.

**Table 1:** Association between PTPRH expression and clinicopathological features of LUAD from TCGA database.

	Low PTPRH	High PTPRH	*P* value
	(*n* = 238)	(*n* = 237)	
Age (years)			
Age < 65	103 (43.3%)	107 (45.1%)	0.75
Age ≥ 65	135 (56.7%)	130 (54.9%)	
Gender			
Female	135 (56.7%)	119 (50.2%)	0.183
Male	103 (43.3%)	118 (49.8%)	
T			
T1	94 (39.5%)	68 (28.7%)	0.0073
T2	124 (52.1%)	127 (53.6%)	
T3	14 (5.9%)	30 (12.7%)	
T4	6 (2.5%)	12 (5.1%)	
N			
N0	168 (70.6%)	145 (61.2%)	0.194
N1	39 (16.4%)	51 (21.5%)	
N2	30 (12.6%)	40 (16.9%)	
N3	1 (0.4%)	1 (0.4%)	
Stage			
Stage I	143 (60.1%)	113 (47.7%)	0.0335
Stage II	53 (22.3%)	64 (27.0%)	
Stage III	35 (14.7%)	45 (19.0%)	
Stage IV	7 (2.9%)	15 (6.3%)	

**Table 2:** Univariate Cox analysis of prognostic factors in LUAD patients.

Id	HR	HR.95L	HR.95H	*P* value
Age	1.193047484	0.883649444	1.610777112	0.249159566
Gender	1.098556611	0.814786594	1.481156707	0.537554253
Stage	1.600081853	1.38591159	1.847348673	1.44E-10
T	1.500920084	1.248216603	1.804783796	1.58E-05
N	1.639585151	1.379833877	1.94823414	1.93E-08
PTPRH	1.124095112	1.048371343	1.205288403	0.001010737

**Table 3:** Multivariate Cox analysis of prognostic factors in LUAD patients.

Id	HR	HR.95 L	HR.95H	*P* value
Age	1.251866713	0.924657859	1.694865026	0.146162723
Gender	1.004833487	0.738891714	1.366492977	0.975475925
Stage	1.388618987	1.115780912	1.72817322	0.003265939
T	1.186372412	0.972206147	1.447717137	0.092478399
N	1.165034604	0.915605604	1.482412975	0.213987103
PTPRH	1.103558766	1.027938508	1.184742026	0.00651251

## Data Availability

The data used to support the findings of this study are provided in the original data. The data and materials in the current study are available from the corresponding author on reasonable request.
